# SALL4 as an Epithelial-Mesenchymal Transition and Drug Resistance Inducer through the Regulation of c-Myc in Endometrial Cancer

This article has been retracted.

**DOI:** 10.1371/journal.pone.0138515

**Published:** 2015-09-25

**Authors:** Lei Liu, Jing Zhang, Xiaoming Yang, Chi Fang, Huali Xu, Xiaowei Xi

**Affiliations:** 1 Department of Obstetrics and Gynecology, Ren Ji Hospital, School of Medicine, Shanghai Jiao Tong University, Shanghai, China; 2 Department of Obstetrics and Gynecology, Shanghai Jiao Tong University Affiliated First People’s Hospital, Shanghai, China; University of Texas Health Science Center, UNITED STATES

## Abstract

SALL4 plays important roles in the development and progression of many cancers. However, the role and molecular mechanism of SALL4 in endometrial cancer remain elusive. In the present research, we have demonstrated that the expression of SALL4 was upregulated in endometrial cancer and correlated positively with tumor stage, metastases and poor survival of patients. The overexpression of SALL4 promoted the invasiveness in endometrial cancer cells, as indicated by the upregulation of mesenchymal cell marker N-cadherin and downregulation of the epithelial marker E-cadherin, and invasion assays in vitro. Additionally, there was also an increase in drug resistance in these cell models due to the upregulation of ATP-binding cassette multidrug transporter ABCB1 expression. Moreover, we also found that ABCB1 was critical for SALL4-induced drug resistance. In contrast, SALL4 knockdown restored drug sensitivity, reversed EMT, diminished cell metastasis and suppressed the downregulation of E-cadherin and the upregulation of N-cadherin and ABCB1. Furthermore, we showed that SALL4 upregulated c-Myc expression and c-Myc was a direct target for SALL4 by ChIP assay, depletion of c-Myc with siRNA abolished the SALL4-induced downregulation of E-cadherin, upregulation of N-cadherin and ABCB1, suggesting that c-Myc was a downstream target for SALL4 and required for SALL4-induced EMT, invasion and drugs resistance in endometrial cancer cells. These results indicated that SALL4 could induce EMT and resistance to antineoplastic drugs through the regulation of c-Myc. SALL4 and c-Myc may be novel therapeutic targets for endometrial cancer.

## Introduction

Endometrial cancer is the seventh most common malignancy with nearly 200000 women diagnosed worldwide every year [1]. In Europe, there are approximately 9000 women dying from endometrial cancer each year. Early diagnosis and treatment have no significant effect on mortality [2]. Surgery, chemotherapy and adjuvant radiotherapy are the main therapeutic methods to endometrial carcinoma. Nevertheless, a minority of patients are sensitive to these therapies [3]. Therefore, it is imperative to find new therapeutic targets to elaborate the molecular mechanisms underlying endometrial carcinogenesis.

SALL4, a member of the SALL gene family, is a transcription factor. It is an essential factor in the maintenance of pluripotency and self-renewal in embryonic stem cells [4–6]. The previous researches have demonstrated that SALL4 participated in regulating the proliferation of hematopoietic stem cells [7, 8]. SALL4 has been shown to participate in the maintenance of chemosensitivity through regulating the ATP-binding cassette (ABC) drug transporter in leukemia [8–10]. The aberrant expression of SALL4 was found in many cancers, including germ cell tumors [11], breast cancer [12], hepatocellular carcinoma [13, 14], gastric cancer [15]. However, the functional role and molecular mechanism of SALL4 are not well characterized in endometrial cancer.

EMT is a fundamental biological process in which epithelial cells undergo a dramatic remodeling of the cytoskeleton, lose basal-apical polarity and acquire an increased capacity to metastasize to distant organs [16–18]. Myometrial invasion is one of the most important prognostic factors in endometrial carcinoma [19]. However, EMT has been poorly understood in endometrial cancer relative to other types of cancer [20].

Multidrug resistance is a common phenomenon in almost all cancers and a major obstacle to successful chemotherapy [21]. Major mechanisms of drug resistance were closely related to the ABC multidrug transporters activated. The ABC multidrug transporters such as ABCB1, ABCC1 and ABCG2 were considered to be responsible for the majority of drug efflux in human cancer [21, 22]. A rise in ABC transporters expression had something to do with a poor prognosis in many types of cancer. ABCB1, also named MDR1, was one of the earliest ABC transporters to be identified. The high expression of ABCB1 was found in the majority of endometrial cancer tissues [23]. Nevertheless, the exact role for ABCB1 in endometrial cancer has not yet been elucidated.

c-Myc oncogene encoded an evolutionarily conserved basic transcription factor, and the expression of c-Myc was commonly aberrant in many cancers [24, 25]. The overexpression of c-Myc has been found to be involved in differentiation, initiation and progression in endometrial cancer [26]. Many studies have demonstrated that the overexpression of c-Myc was closely linked to chemotherapy resistance and EMT process. Therefore, we are interested in determining whether c-Myc is involved in chemotherapy resistance and EMT in endometrial cancer.

In the present research, we demonstrated that SALL4 expression was upregulated and associated with poor survival in endometrial cancer. SALL4 in endometrial cancer cells not only induced the acquisition of properties of EMT, but also promoted migration and invasion through the activation of c-Myc. In addition, we also found that c-Myc served as a direct target gene of SALL4 and was involved in SALL4-induced drug resistance by regulating the expression of ABCB1. In conclusion, these findings indicate that SALL4 plays important roles in endometrial cancer metastasis and drugs resistance, with c-Myc as a major downstream target.

## Materials and Methods

### Patients and tissues

80 endometrial cancer specimens and 10 normal endometrial samples were obtained from patients who underwent surgical treatment from 2010 to 2013 at the Shanghai Jiao Tong University Affiliated Shanghai First People's Hospital (Shanghai, China). Another six pairs of frozen nontumorous tissues and matched adjacent endometrial cancer tissues were obtained from six patients at Shanghai First People's Hospital from 2014 to 2015. No patient had received neoadjuvant therapy before the surgery. Written informed consent was obtained from all patients. The Human Investigation Ethical Committee of Shanghai First People's Hospital Affiliated Shanghai Jiao Tong University approved this study.

### Cell culture

Endometrial cancer cell lines RL95-2, Ishikawa, HEC1-A, HEC1-B, AN3CA and KLE were obtained from the Chinese Academy of Sciences Committee Type Culture Collection (Shanghai, China). Cells were cultured in DMEM added with 10% fetal bovine serum.

### Immunohistochemistry

Immunohistochemistry was carried out on paraffin-embedded tissues using primary antibodies as follows: anti-SALL4 (Santa Cruz Inc., Santa Cruz, CA, USA). For assessment of the expression of SALL4, staining intensity was scored as 3 (strong), 2 (medium), 1 (weak), or 0 (negative). The degree of staining was scored as 4 (76%–100%), 3 (51%–75%), 2 (26%–50%), 1 (1%–25%), or 0 (0%). The sum of the extent score and the intensity score was regarded as the final staining score. A final staining score ≥ 4 was positive for expression.

### Knockdown of SALL4 in AN3CA cells

The high SALL4 expression endometrial carcinoma cell line AN3CA was used to establish the stable SALL4 knockdown cell line. SALL4-shRNA1 and SALL4-shRNA2 lentiviral plasmids (GenePharma, Shanghai, China) were used to perform the knockdown experiment. AN3CA cells infected with a scrambled shRNA were regard as a control. SALL4 knockdown efficiency was confirmed by western blotting. The sequences for scrambled shRNA and SALL4 shRNAs are listed as following: SALL4shRNA1:5'GCCTTGAAACAAGCCAAGCTA3';SALL4shRNA2:5'CTATTTAGCCAAAGGCAAA3' and Scr-shRNA: 5'CCTAAGGTTAAGTCGCCCTCG3'.

### Transfection

Plasmid construction were performed in accordance with standard procedures. For cloning of SALL4A (GenBank accession no. AY172738) and SALL4B (GenBank accession no. AY170621) isoforms, polymerase chain reaction (PCR) primers were designed. SALL4A and SALL4B cDNA in an expression vector were synthesized from GenePharma (Shanghai, China). Ishikawa cells were stably transfected with SALL4A or SALL4B. The sequences for c-Myc siRNA: Sense: 5'-GGACUAUCCUGCUGCCAAGdTdT-3', Antisense:3'-dTdT CCUGAUAGGACGACGGUUC-5'. The sequences for ABCB1 siRNA: Sense: 5'-AGAGAAGAAACCAGUGGUC-3', Antisense: 5'-GACCACUGGUUUCUUCUCU-3'. According to the protocol of the manufacturer, siRNA were transfected by using Lipofectamine 2000 (Invitrogen).

### Western blotting

Western blotting was performed as described previously [27]. In brief, proteins were extracted from cultured cells and separated by SDS-PAGE. Proteins of interest were determined using corresponding specific antibodies after transferring to PVDF membranes. The following antibodies were used for analysis: antibody against c-Myc (Rabbit polyclonal, Cell Signaling (Beverly, MA, USA); D84C12), anti- SALL4 (mouse monoclonal, Santa Cruz Inc, SC-101147) and anti-ABCB1 (mouse monoclonal, Santa Cruz Inc, SC-55510). Anti-E-cadherin (Rabbit Polyclonal, ab53226), anti-N-cadherin (Rabbit Polyclonal, ab18203) and GAPDH (Rabbit monoclonal, ab181603) were purchased form Abcam (Cambridge, UK).

### Quantitative RT-PCR

According to the manufacturer’s instructions, total RNA was prepared using TRIzol (Invitrogen) and reverse transcribed as previously described [28]. Primers for ABCB1, E-cadherin, N-cadherin, c-Myc and GAPDH genes were synthesized from Invitrogen Bioengineering Corporation (Shanghai, China). qRT-PCR reactions were set up with 2μl cDNA template, 10μl SYBR Green PCR Master Mix and 1μl primer mixture. The PCR conditions were 95°C for 5 min, followed by 40 cycles of 94°C for 1 min, 60°C for 30 s and 72°C for 45 s.

### Chromatin immunoprecipitation

According to the manufacturer’s protocol, the ChIP assay was carried out by the use of the ChIP-IT kit (Active Motif). Chromatinimmunoprecipitated DNA was subjected to PCR amplification for the SALL4 binding site in the promoter of c-Myc. Specific c-Myc primers are as follows: forward: 5'-TCAAGAGGCGAACACACAAC-3'; reverse: 5'-GGCCTTTTCATTGTTTTCCA-3'. The PCR product (c-Myc: 110bp) was resolved by electrophoresis in a 1% agarose gel and visualized by ethidium bromide staining.

### Cell viability assay

A different concentration of carboplatin (0, 20, 40 and 60μg/ml) treated cells plated in 96-well plates. Cell Counting Kit-8 (Dojindo, Japan) was used to assess cell viability after treating with carboplatin for 24 h. The absorbance was examined at 450 nm through a microplate reader.

### Colony formation assay

About 10^3^ cells were plated in a six-well culture plate. Cells were fixed with 10% formaldehyde solution and stained with 10% Giemsa after treating with 20μg/ml carboplatin at 37°C incubator for 10 days. The number of colonies containing >50 cells was counted under a microscope.

### Wound-healing assay

A scratch was drawn into the cell layer after 24 h of incubation in a 6-well plate. Photographs were taken at 0 h and 48 h to measure the migration. The distance of cells migration was examined.

### Cell invasion assay

1×10^5^ cells were seeded in the upper chamber of 24-well transwell plates (Corning, NY, USA) coated with BD matrigel basement membrane matrix with serum-free medium. DMEM/F12 supplemented with 10% fetal bovine serum was added to the lower chamber. After incubating for 16 h, the invasive cells were counted under a microscope. All the samples were plated in triplicate.

### Statistical analyses

All the data are presented as mean ± standard deviation. Statistical significance was analyzed by Student’s t-test. Chi square test for 2×2 tables was used to compare categorical data. The value of P<0.05 was considered significant. All experiments were performed in triplicate.

## Results

### The expression of SALL4 is upregulated and associated with poor survival in endometrial cancer

To identify the function of SALL4 in endometrial cancer, we firstly assessed the expression of SALL4 in six fresh nontumorous tissues and matched adjacent endometrial cancer tissues. As shown in Fig 1A, SALL4 expression in endometrial cancer tissues was significantly higher than that in nontumorous tissues (P<0.05). The expression of SALL4 in 80 endometrial cancer tissues and 10 normal endometrial tissues was examined through immunohistochemistry. We found that SALL4 was higher in endometrial cancer (56/80) compared with normal endometrial tissues (0/10) (Fig 1B, S1 Table). The difference was statistically significant in the two groups (P<0.01). The association between the expression of SALL4 and clinicopathological characteristics was showed in Table 1. We showed that an increased SALL4 expression in endometrial cancer was significantly associated with lymph node metastasis (P = 0.048), tumor stage (P = 0.001), myometrial invasion (P = 0.007) and poor survival (Fig 1C). In conclusion, these results indicate that SALL4 expression in endometrial cancer is closely related to poor survival of patients.

**Fig 1:** SALL4 expression is upregulated in endometrial cancer and associated with poor prognosis. (A) The expression of SALL4 in endometrial cancer tissues and nontumorous tissues was assessed through western blotting. (B) The images showed immunohistochemical staining of SALL4 in normal endometrium and endometrial cancer tissues (00D7200). (C) Kaplan-Meier analysis indicated that the expression of SALL4 was associated with poor survival of patients.

**Table 1:** Relationship between SALL4 expression and clinicopathologic characteristics in endometrial cancer (n = 80).

Parameter	N	Positive (%)	*P*
Age			
≤50	33	22 (66.7%)	0.586
>50	47	34 (72.3%)	
FIGO stage			
I-II	52	30 (57.7%)	0.001
III-IV	28	26 (92.9%)	
Histological grade			
G1	38	29 (76.3%)	0.309
G2	29	20 (69.0%)	
G3	13	7 (53.9%)	
Lymph node metastasis			
Positive	26	22 (84.6%)	0.048
Negative	54	34 (63.0%)	
Myometrial invasion			
≤1/2	45	26 (57.8%)	0.007
>1/2	35	30 (85.7%)	

### SALL4 induces the EMT and invasive phenotype in endometrial cancer cells

We wanted to determine whether SALL4 was involved in EMT and metastasis among endometrial cancer cells, SALL4 expression was evaluated to choose appropriate cell lines for our research in endometrial cancer cell lines: AN3CA, KLE, HEC1-B, HEC1-A, RL-952 and Ishikawa. As shown in Fig 2A, AN3CA and KLE cells showed obvious mesenchymal phenotype, but Ishikawa and RL-952 cells showed apparent epithelial characteristics (S1 Fig). The expression of SALL4 was associated with the epithelial/mesenchymal characteristics in these endometrial cancer cell lines. Cells associated with relatively strong mesenchymal characteristics showed a high SALL4 expression. Two shRNAs specifically targeting both SALL4A and SALL4B were used to knock down endogenous SALL4 in AN3CA cells with relatively higher expression of SALL4. Knockdown of SALL4 protein levels in AN3CA cells led to increased protein and mRNA levels of the epithelial label E-cadherin and decreased that of the mesenchymal marker N-cadherin, accompanying with cells morphological transition from a scattered spindle-shaped mesenchymal appearance to a round, tightly packed morphology (Fig 2B, 2C and 2D). In addition, knockdown of SALL4 (Fig 2E and 2F) in AN3CA cells attenuated cell migration and invasion ability. On the contrary, Ishikawa cells with low endogenous level of SALL4 were transfected with SALL4A and SALL4B cDNA vector (Control vector). Overexpression SALL4 led to a morphological change from a tightly packed, round morphology to a spindle-shaped scattered morphology in Ishikawa cells, decrease protein and mRNA levels of the epithelial label E-cadherin and increase that of the mesenchymal marker N-cadherin (Fig 2B, 2C and 2D). Overexpression of SALL4 dramatically increased migration and invasion ability of Ishikawa cells (Fig 2E and 2F). In brief, these data suggest that SALL4 induces the EMT and metastasis in endometrial cancer cells.

**Fig 2:** SALL4 induces the EMT and invasive phenotype in endometrial cancer cells. (A) N-cadherin, E-cadherin, SALL4A and SALL4B were assessed by western blotting in endometrial cancer cell lines: AN3CA, KLE, HEC1-B, HEC1-A, RL-952 and Ishikawa. (B) Cell morphology was examined in Ishikawa cells transfected with SALL4A or SALL4B expression vector and AN3CA cells transfected with SALL4-sh1 or SALL4-sh2. (C)(D) The protein and mRNA levels of E-cadherin and N-cadherin were analyzed in Ishikawa cells transfected with SALL4A or SALL4B expression vector and AN3CA cells transfected with SALL4-sh1 or SALL4-sh2. (E) Cell migration and invasion of Ishikawa or AN3CA were examined through wound healing assay and transwell invasion assay. (F) The degree of migration and invasion in Ishikawa and AN3CA cells was analyzed. *P<0.01.

### SALL4 drives chemotherapeutic drug resistance in endometrial cancer cells

Drug resistance is a significant obstacle that affects the overall survival rate for advanced and recurrent endometrial cancer patients. We sought to test whether SALL4 in endometrial cancer cells participated in mediating cellular resistance to chemotherapeutic drugs. It was revealed by cell viability assay that an increase in cell viability upon exposure to carboplatin was much more pronounced in Ishikawa cells transfected with either SALL4A or SALL4B than in cells transfected with empty vector (Fig 3A). Meanwhile, overexpression SALL4 in the role of cells proliferation was examined through clone formation assay in Ishikawa cells treated with 20μg/ml carboplatin. Ishikawa cells transfected with SALL4A or SALL4B displayed increased carboplatin resistance and cell proliferation compared with control (Fig 3B). On the contrary, cell viability assay and clone formation assay indicated that knockdown of SALL4 significantly reduced resistance to carboplatin in AN3CA cells (Fig 3A and 3B). In summary, these findings indicate that SALL4 induces drug resistance in endometrial cancer cells.

**Fig 3:** SALL4 drives endometrial cancer cells chemotherapeutic drug resistance. (A) Ishikawa cells transfected with SALL4A or SALL4B expression vector and AN3CA cells transfected with SALL4-sh1 or SALL4-sh2 were treated with the indicated concentrations of carboplatin, and cell viability assay were performed. (B) Ishikawa cells transfected with SALL4A or SALL4B expression vector and AN3CA cells transfected with SALL4-sh1 or SALL4-sh2 were treated with carboplatin, clone formation assay were performed. **P<0.01, *P<0.05.

### ABCB1 is critical for SALL4-induced drug resistance

The majority of drug resistance in human cancer are associated with ATP-binding cassette (ABC) multidrug transporters. It is not clear whether ABCB1 is involved with SALL4-induced chemotherapy resistance and a downstream target gene directly regulated by SALL4 in endometrial cancer. It was revealed through western blotting that SALL4 upregulation in SALL4A- or SALL4B-transfected Ishikawa cells significantly increased the protein expression of ABCB1 compared with empty vector (Fig 4A). A similar SALL4 knockdown experiment was put into effect in AN3CA cells. As shown in Fig 4A, SALL4 silencing could apparently decrease ABCB1 protein expression. These data indicated that SALL4 could upregulate the expression of ABCB1. Because ABCB1 (MDR1) was essential for drug resistance and upregulated in endometrial cancer, we wanted to determine whether ABCB1 was involved in SALL4-induced drug resistance. We further silenced ABCB1 expression by specific siRNA in Ishikawa cells overexpressing SALL4, and found that downregulation of ABCB1 reduced SALL4-induced drug resistance (Fig 4B and 4C). The downregulation of the mRNA and protein levels of ABCB1 was confirmed by qRT-PCR and western blotting (Fig 4D and 4E). Taken together, these data demonstrate that SALL4 induces chemotherapeutic drug resistance through the regulation of ABCB1 in endometrial cancer cells.

**Fig 4:** ABCB1 is critical for SALL4-induced drug resistance. (A) Western blotting showed that ectopic overexpression of SALL4 upregulated ABCB1 protein expression in Ishikawa cells and knockdown of SALL4 in AN3CA cells downregulated ABCB1 expression. (B)(C) Ishikawa cells transfected with SALL4A or SALL4B vector or control vector were transfected with si-ABCB1 or control siRNA. Drug sensitivity of Ishikawa cells to carboplatin was examined by cell viability assay and clone formation assay. (D)(E) The protein and mRNA levels of ABCB1 were assessed by western blotting and qRT-PCR. **P<0.01.

### c-Myc is required for SALL4-induced EMT and drug resistance

c-Myc plays important roles in many oncogenic processes, including tumor drug resistance and metastasis. The previous research has shown that SALL4 in endometrial cancer cells promoted c-Myc transcriptional activity [29]. We were interested in determining whether c-Myc was required for SALL4-induced EMT and chemotherapy resistance. Consistent with the previous study, we showed that the expression of c-Myc was positively correlated with that of SALL4 by western blotting, and c-Myc was a direct target of SALL4 through ChIP assay in endometrial cancer cells (Fig 5A, 5B and S2 Fig). We next silenced c-Myc expression by siRNA in SALL4A- and SALL4B-transfected Ishikawa cells, and showed that c-Myc downregulation dramatically reduced SALL4-induced cell invasion and drug resistance (Fig 5C, 5D and 5E). The protein and mRNA levels of c-Myc were detected by western blotting and qRT-PCR (Fig 5F and 5G). Moreover, the reversal of the invasive phenotype induced by c-Myc silencing in SALL4 overexpression in Ishikawa cells was confirmed by downregulation of mesenchymal marker N-cadherin and upregulation of epithelial marker E-cadherin by western blotting and qRT-PCR (Fig 5F and 5H). At the same time, we also found that c-Myc siRNA treatment significantly diminished SALL4-induced ABCB1 protein level (Fig 5F). These results indicate that c-Myc is required for SALL4-induced EMT and chemotherapy resistance.

**Fig 5:** c-Myc is required for EMT and chemotherapy resistance by SALL4-induced. (A) The expression of c-Myc was positively associated with that of SALL4 in Ishikawa and AN3CA cells by western blotting analysis. (B) c-Myc was a direct target of SALL4 through ChIP assay. (C) Downregulation of c-Myc by specific siRNA reduced SALL4-induced invasion in Ishikawa cells overexpressing SALL4 by transwell assay. (D)(E) Downregulation of c-Myc reduced SALL4-induced drug resistance in Ishikawa cells overexpressing SALL4 through viability assay and clone formation assay. (F) The expression of EMT-related markers and ABCB1 was assessed by western blotting in Ishikawa cells. (G)(H) The mRNA levels of c-Myc, E-cadherin and N-cadherin were detected through qRT-PCR in Ishikawa cells. **P<0.01.

## Discussion

It is becoming increasingly clear that aggressive tumor cells show a plastic, multipotent phenotype similar to the pluripotent/stem-like state in embryonic cells and basal-like tumor cells [30]. The embryonic stem cell-like gene expression signature has been demonstrated to be closely related to poorly differentiated aggressive human tumors and has been regarded as a potential target for future cancer therapies [31]. SALL4 is a transcription factor that maintains pluripotency and self-renewal in embryonic stem cells and plays an important role in embryonic development. However, the functional roles and molecular mechanism of SALL4 in endometrial cancer are not well characterized.

In the present study, we demonstrated that SALL4 expression was upregulated in endometrial cancer and positively correlated with poor prognosis and aggressive properties. We showed that an increased expression of SALL4 promoted metastasis by EMT process as well as chemotherapy resistance through modulating ABCB1 in endometrial cancer cells. Significantly, we found that a downstream target of SALL4, c-Myc, was indispensable to SALL4-induced EMT and the expression of ABCB1. These findings revealed that SALL4 and c-Myc might be promising therapeutic targets in endometrial cancer (Fig 6).

**Fig 6:** Schematic diagram of the c-Myc-mediated SALL4-induced EMT and chemoresistance signaling pathways in endometrial cancer cells. SALL4 induced EMT and ABCB1 expression, which subsequently contributed to invasion and chemoresistance in endometrial cancer cells. ABCB1 was critical to SALL4-induced chemoresistance. In addition, SALL4 also upregulated c-Myc expression, which was required for SALL4-induced EMT and ABCB1 expression. In summary, SALL4-induced EMT and drug resistance through the activation of c-Myc in endometrial cancer.

SALL4 plays important roles in multiple tumor-associated processes, including cell metastasis and drug resistance. Metastasis is not only the main cause of cancer death but also the malignant properties of cancer. Cancer cells which undergo EMT process will acquire the invasiveness and metastasis ability. The present research showed that SALL4 induced EMT-related proteins including a decrease in cellular adhesion molecules E-cadherin and an increase in mesenchymal marker N-cadherin. The expression of E-cadherin and N-cadherin was closely associated with cancer cells invasive and metastatic capacity. Our results were supported by the previous studies showing that the downregulated expression of E-cadherin was significantly associated with myometrial invasion and patient survival in endometrial carcinoma [32, 33]. The recent researches have shown that SALL4 was involved in the metastasis and progression in colorectal cancer [34]. In addition, SALL4 overexpression induced EMT in gastric cancer cells, with increased expression of Twist1, N-cadherin and decreased expression of E-cadherin [15]. Meanwhile, it was reported that SALL4 suppressed the expression of adhesion gene CDH1 (E-cadherin), and positively regulated the CDH1 suppressor ZEB1 and maintained cell dispersion in basal-like breast cancer [35]. This evidence suggested that SALL4 could induce EMT and promote invasion in a variety of tumors. In agreement with a previous study [29], we found that upregulation of SALL4 significantly increased endometrial cancer cells migration and invasion. More importantly, we demonstrated that overexpression SALL4 was able to induce EMT and promote metastasis in endometrial cancer cells.

Chemotherapeutics is the most effective treatment for patients with metastatic cancer. However, drug resistance remains a serious impediment to successful chemotherapy [21]. Among various mechanisms involved in chemotherapeutic resistance, ABC transporters were thought to be closely related to drug resistance. Mounting evidence indicated that ABC transporters played important roles in SALL4-induced chemotherapeutic resistance in a variety of cancers. For example, it was recently reported that SALL4 was involved in chemotherapeutic resistance by directly regulating the downstream target gene ABCA3 in acute myeloid leukaemia [10]. Moreover, recent reports have shown that SALL4 positively regulated the expression of ABCA3, affecting the sensitivity to chemotherapy drug in chronic myeloid leukaemia [36]. Overexpression of SALL4 led to an increased cell proliferation associated with the upregulated expression of (ATP)-binding cassette-G2 (ABCG2) in hepatocellular carcinomas [13]. ABCB1 is the prototype of this gene superfamily, and its deregulation has been associated with drug resistance in several types of cancers [21]. Evidence had shown that the expression of ABCB1 was abnormal in endometrial carcinoma [23]. These findings prompted us to investigate whether ABCB1 participated in SALL4-induced chemotherapy resistance in endometrial carcinoma. In accordance with the role of SALL4-induced drug resistance via modulating ABC transporters in other cancers, we found that ABCB1 was involved in SALL4-induced drug resistance in endometrial cancer. Downregulation of ABCB1 significantly blocked SALL4-induced drug resistance. These data suggested that ABCB1 was an important mediator among SALL4-induced drug resistance in endometrial cancer.

The previous study has shown that c-Myc induced EMT in mammary epithelial cells [37]. In addition, c-Myc can contribute to the cancer cells chemoresistant phenotype through regulating ABC transporter genes [38]. It was reported that c-Myc combined with epigenetic mechanisms regulated ABC transporter genes expression in CML [39]. In the present study, we found that c-Myc was a direct target of SALL4 and required for EMT and ABCB1 expression induced by SALL4, leading to metastasis and drug resistance in endometrial cancer cells. It was demonstrated by previous studies that higher expression of c-Myc was significantly associated with decreased overall survival in endometrial carcinoma patients [40, 41]. Moreover, it was also reported that the transcriptional activity of c-Myc was regulated directly by SALL4 in endometrial cancer cells [29]. Our data were in accordance with the previous these results. However, the present study was the lack of data involved in assessing the expression of ABCB1 and c-Myc in endometrial cancer specimens. It would be more convincing if the data that the expression level of SALL4 was positively associated with those of ABCB1 and c-Myc in a subset of endometrial cancer specimens was supplemented. In summary, c-Myc was of the essence in SALL4-induced EMT and drug resistance and might be a therapeutic target for endometrial carcinoma.

Taken together, we demonstrated that SALL4 expression was upregulated in endometrial cancer and positively correlated with poor prognosis and aggressive properties. We identified that SALL4 not only induced EMT, but also increased drug resistance through ABCB1 in endometrial cancer cells. We further showed that c-Myc was indispensable for SALL4-induced EMT and chemotherapy resistance. In conclusion, our study provided a potential molecular mechanisms related to SALL4-induced invasion and chemotherapy resistance in endometrial cancer. SALL4 and c-Myc may be novel therapeutic targets for endometrial cancer.

## Supporting Information

S1 Fig SALL4 induces EMT in endometrial cancer cells. (A) The mRNA level of E-cadherin and N-cadherin was assessed through qRT-PCR in endometrial cancer cell lines: AN3CA, KLE, HEC1-B, HEC1-A, RL-952 and Ishikawa.
(TIF)

S2 Fig c-Myc is a target for SALL4 in endometrial cancer cells. Chromatinimmunoprecipitated DNA was assessed through quantitative PCR in endometrial cancer cells AN3CA and Ishikawa.
(TIF)

S1 Table SALL4 immunohistochemical staining score in endometrial cancer. (DOCX)
